# *MCM6* Promotes Hepatocellular Carcinoma Progression via the Notch Pathway: Clinical, Functional, and Genomic Insights

This article has been retracted.

**DOI:** 10.1155/2022/3116303

**Published:** 2022-06-09

**Authors:** Liangjuan Hou, Xin Zeng, Xuan Li, Chune Zhao, Juan Zou, Yukun Li, Gang Liu

**Affiliations:** ^1^Department of Histology and Embryology, Chongqing Three Gorges Medical College, Wanzhou, Chongqing 404120, China; ^2^Department of Embryo Laboratory, Changsha Reproductive Medical Hospital, Changsha, Hunan 410000, China; ^3^Department of Infectious Disease, Three Gorges Hospital of Chongqing University, Chongqing University, Wanzhou, Chongqing 404000, China; ^4^Hunan Province Key Laboratory of Tumor Cellular & Molecular Pathology, Cancer Research Institute, University of South China, Hengyang, Hunan 421001, China

## Abstract

**Objective:**

To evaluate the expression profile of MCM6 in HCC and the relationship between MCM6 level and clinicopathological parameters through bioinformatics analysis of several databases.

**Methods:**

MCM expression level, clinical parameters, survival data, and gene set enrichment analysis were analyzed by bioinformatics database, including Oncomine™, UALCAN, HCCDB, TCGA, cBioPortal, and LinkedOmics. Real-time PCR, western blotting, and IHC staining were conducted to identify the expression of *MCM6* in HCC compared to normal liver tissues.

**Results:**

Bioinformatics analysis indicated that the mRNA of *MCM6* was obviously increased in multiple cancer types, especially in HCC. *MCM6* level was positively associated with multiple clinical parameters (stage 3 and grades 3 and 4) and negatively associated with patient outcomes (overall survival). Moreover, enrichment of functions and signaling pathways analysis of *MCM6* suggested that *MCM6* might mediate DNA replication and cellular metabolism to promote the development and progression of HCC. Furthermore, IHC staining and western blotting indicated that the *MCM6* was enhanced in HCC tissue, and *MCM6* could promote HCC proliferation in activating Notch pathway via WB and bioinformatic analysis.

**Conclusion:**

This study actually revealed the expression and related functions of *MCM6* in HCC. Furthermore, *MCM6* is a carcinogenic role in activating Notch pathway to promote HCC cell proliferation, which may be a new prognostic biomarker and therapeutic target for HCC patients.

## 1. Introduction

Hepatocellular carcinoma (HCC) is the sixth most lethal human malignancy globally, with 841,080 new and 781,631 deaths cases estimated for 2018 [1]. The World Health Organization has predicted that more than 1 million people will die from HCC in 2030 [2]. Moreover, the incidence and death rates of HCC are increasing in developing countries [3]. Despite the improvements in surgery combined with radiotherapy and chemotherapy, the high mortality and low 5-year survival rate of HCC are primarily due to the complex pathophysiological processes, including hepatitis, liver fibrosis, and abnormal regeneration of liver cells. Identifying key multigene networks in multiple steps is necessary to enhance the early metaphase diagnosis rate [2]. Early diagnosis of HCC may be able to prolong the lifespan of patients with HCC as much as possible [4]. Therefore, it is of great clinical significance to explore accurate biomarkers for early diagnosis and potential treatment targets in HCC.

Minichromosome maintenance (MCM) proteins family, a classical family on the eukaryotic genome replication, in Saccharomyces cerevisiae, was found first, which were necessary for the maintenance of extrachromosomal DNA [5]. During the DNA replication licensing process, *MCM2*-7 forms a hexameric ring-shaped complex to promote DNA replication of chromatin by binding to a DNA replication starting point in the middle to late cell cycle to the early G1 phase [6]. A biochemical and structural study indicated that the hexameric ring-shaped complex was a hetero-hexameric AAA+ ATPase, which has helicase activity, while the N-terminal region plays the role of organizing center in the replication in eukaryotic cells [7].

*MCM6*, as an important member of the MCM family, could interact with Cdt1 at NTD to stabilize the coil structure [8], be phosphorylated by *DDK* at NTD terminus to activate pre-RC [9], and be involved in translocation along single-stranded DNA in the *MCM2*-7 complex [8]. It is reported that *MCM6*, as a transcriptional regulation factor, could activate *MEK/ERK* signaling pathway to mediate EMT progression, resulting in metastasis of HCC [10]. Chen et al. [11] found that the direct interaction between *MCM6* and p53-binding protein 1 (*53BP1*) was involved in *53BP1* chromatin fraction and foci formation in HepG2 cells. However, little is known about the role and mechanism of *MCM6* in hepatocarcinogenesis. Until now, the previous studies indicated that the expression of *MCM6* was observed in 70 patients with HCC, and it may relate to poor prognosis [10].

This study evaluated the expression profile of *MCM6* in HCC and the relationship between *MCM6* level and clinicopathological parameters through bioinformatics analysis of several databases. In addition, the biological functions and genomic changes correlated with biological functions in HCC were examined. The present study may provide a novel and potential molecule target for the early diagnosis and targeted therapy of HCC.

## 2. Materials and Methods

### 2.1. Bioinformatic Analysis

Oncomine database (http://www.oncomine.org) is a web tool to extract data for the mRNA level and gene expression of *MCM6*, currently containing 715 datasets and 86,733 samples. A series of HCC datasets were utilized for this study, including Chen Liver, Roessler Liver, and Roessler Liver 2. HCCDB database (http://lifeome.net/database/hccdb/search.html) is an integrative molecular database of HCC based on 4000 HCC samples. We utilized the HCCDB database to confirm the level of *MCM6*. UALCAN database (http://ualcan.path.uab.edu) is an interactive web portal to analyze the expression of *MCM6* in HCC, which is based on gene expression analysis of TCGA (The Cancer Genome Atlas). The cBioPortal database (http://cbioportal.org) is an interactive web tool for elucidating the altered expression of *MCM6*, which is used to explore the multidimensional genomics datasets for multiple cancer types. LinkedOmics database (http://www.linkedomics.org/login.php), as an online tumor database, was utilized for elucidating multiomics data. Users can extract multiple cancer-type protein expression profiles, which are differential expression in specific cancer. We used it to analyze the GO and KEGG pathway of *MCM6* coexpression genes in HCC.

### 2.2. Cell Culture and Tissue Collection

Two HCC cell lines (HepG2 and SNU-368) were cultured in Dulbecco's Modified Eagle Medium (DMEM; Gibco) containing 10% fetal bovine serum (FBS) and 100 U/mL penicillin and streptomycin, which were maintained at 37°C in a humidified atmosphere of containing 5% CO_2_. Furthermore, a total of 30-paired HCC and paracancerous tissues were surgically obtained from the Three Gorges Hospital of Chongqing University in Wanzhou, China. This study was approved by the ethics committee of Three Gorges Hospital of Chongqing University with the written consent of all patients.

### 2.3. Cell Transfection

The shRNA against *MCM6* or shRNA negative control were constructed by RiboBio Co. Ltd. siRNA was transfected into cells using riboFECT transfection reagent (Changzhou Bio-Generating Biotechnologies Co., Ltd.) according to the manufacturer's protocol. The sequences of the siRNA were as follows: si-*MCM6*, GGCGCATAGTAGATTTGCA. The shRNAs were transfected by lip3000 for 6 hours. The effect of MCM6 knockdown was confirmed by western blot.

### 2.4. Western Blot

Western blotting was conducted according to our previous report [12]. The experiment was conducted with the approval of a formal Ethics committee and the informed consent of the patients. The primary antibodies were used in this study against *MCM6* (ab201683, dissolution 1/1000), NICD (Santa Cruz, sc6014, dissolution 1/500), *Notch1* (ab52627, dissolution 1/1000), *Hey1* (ab154077, dissolution 1/1000), *Hes1* (ab119776, dissolution 1/1000), and *GAPDH* (ab181603, dissolution 1/10000).

### 2.5. Immunohistochemistry Analysis

The slices are dewaxed and then hydrated. After blocking endogenous peroxidase, the slices were treated with a hot citric acid buffer to reveal the epitope. The sections were then incubated with a primary antibody using an immunohistochemistry kit (MXB, Fuzhou, China) according to the manufacturer's instructions.

Immunohistochemical staining scores were assessed by staining percentage of tumor cells and staining intensity. The percentage of stained cancer cells was graded from 0 to 4: 0 (0% stained), 1 (0%-25% stained), 2 (26%-50% stained), 3 (51%-75% stained), and 4 (76%-100% stained). Similarity, stained tumor cell intensity was divided into 0 (negative), 1 (weak), 2 (moderate), and 3 (strong). The final semi-quantitative immunohistochemical fraction was obtained by multiplying the percentage of stained cancer cells by the intensity grade.

### 2.6. Proliferation Analysis

For the MTT analysis, two HCC cancer cell lines were seeded in 96-well (5 × 10^3^) and cultured for one, two, and three days. 20 *μ*l MTT solution (Sigma-Aldrich; Merck KGaA) was used to incubate for 2 hours. Next, 150 *μ*l DMSO was added in each well. Last, the OD value was confirmed at 490 nm by a microplate reader. For the clone formation assay, cells were seeded into 24-well plates with 500 cells in each well and cultured for 14 days.

When cell colonies were visible to the naked eyes, the culture was terminated—washed cells with PBS for 3 times, 5 minutes each time. Then fix with 4% paraformaldehyde for 20 minutes. The cells were washed with PBS for 3 times, 5 minutes each time, incubated with methanol for 20 minutes, and washed with PBS for 3 times, 5 minutes each time. Shake dry and stain with crystal violet for 30 minutes. Take photos and analyze the results.

### 2.7. Statistical Analysis

Statistical analyses for bioinformatic analysis were performed in the R Programming Language (version 3.6). Data are presented as the mean ± SD. All assays were tested in three independent experiments. Experimental data were analyzed using SPSS statistical software (version 12.0; SPSS Inc.). The significance of the group difference was evaluated by one-way analysis of variance followed by Tukey's post hoc test. Multiple comparisons between the groups were performed using Student-Newman-Keuls method. *P* < 0.05 was considered to indicate a statistically significant difference.

## 3. Results

### 3.1. The *MCM6* Level Was Enhanced in HCC

We firstly extracted *MCM6* transcription levels from a variety of cancers from TCGA. The Oncomine database indicated significant increases in *MCM6* mRNA expression in HCC (Figures 1(a) and 1(b)). To further determine the expression of *MCM6* in many cancers, we extracted the expression profile of *MCM6* based on TCGA database. As shown in Figure 2(a), we found *MCM6* transcription expression was obviously enhanced in lung cancer, head and neck squamous cell carcinomas, HCC, and so on. The 4D measurement of the HCCDB dataset showed that *MCM6* was not a liver-specific gene (logFC = −1.58), and *MCM6* were increased in HCC compared to normal liver tissue (logFC = 0.34) and corresponding paracancer tissue (logFC = 0.91) (Figure 1(c)). In addition, high level of *MCM6* was found in a subgroup evaluation of HCC samples with various clinicopathologic features (UALCAN database). *MCM6* profile was obviously increased in tumor grade, cancer stage, patient age, gender, race, and weight (Figures 2(b)–2(g)). In summary, *MCM6* can be used as a possible diagnostic marker for HCC.

### 3.2. *MCM6* Genetic Alteration Correlated with Patient Survival in HCC Patients

In the cBioPortal dataset, we extracted the profile of *MCM6* genetic alteration in HCC. Three HCC databases (AMC hepatology 2014 dataset, INSERM Nat Genet 2015 dataset, TCGA Firehose Legacy dataset) analysis results indicated that the highest alteration frequency of *MCM6* was only 1% (Figures 3(a) and 3(b)). Furthermore, the patients with *MCM6* alteration had significant disease/progression-free survival (Figure 3(d)), but had no significant overall survival (Figure 3(c)). UALCAN analysis suggested that these HCC patients with a high level of *MCM6* had a worse prognosis (Figure 3(e)). Hence, these results indicated that *MCM6* alteration might induce an unfavorable prognosis in HCC patients.

### 3.3. Gene Coexpression of *MCM6* in HCC

The method analyzed mRNA sequencing data from 371 HCC patients by LinkedOmics analysis of genes coexpressed with *MCM6*. The heat map showed the top 50 significant positively and negatively coexpressed genes with *MCM6*, respectively (Figures 4(a) and 4(b)). The volcano blot showed all the coexpressed genes with *MCM6* (Figure 4(c)). For example, *NDUFAF1*, *LDHD*, and *SERPING1* were the most significantly and negatively correlated with the expression of *MCM6* (Figures 5(a)–5(c)), while *DTL*, *ZWINT*, and *MCM2* were the top 3 negatively correlated genes with *MCM6* (Figures 5(d)–5(f)). These genes were involved in many biological progressions, such as cell proliferation, transcription, metastasis, cell cycle, and metabolism. Gene set enrichment analysis (GSEA) was used to analyze GO annotation with significant enrichment. In these differentially expressed genes (DEGs) associated with *MCM6*, the GO enrichment results indicated that (1) for biological process (BP), these DEGs were obviously enriched in biological regulation, metabolic process, response to stimulus, multicellular organismal process, localization, and cellular component organization (Figure 6(a)); (2) for cellular component (CC), these DEGs were significantly enriched in the membrane, nucleus, membrane-enclosed lumen, protein-containing complex, cytosol, endomembrane system, and vesicle (Figure 6(b)); (3) for molecular function (MF), these DEGs were largely enriched in protein binding, ion binding, nucleic acid binding, hydrolase activity, transferase activity, and nucleotide-binding (Figure 6(c)). The signaling pathway enrichment analysis by KEGG showed that these DEGs were primarily enriched in primary bile acid biosynthesis, valine, leucine and isoleucine degradation, arginine biosynthesis, DNA replication, fatty acid degradation, and homologous recombination (Figure 6(d)).

### 3.4. Identification of *MCM6* Expression and Prognosis in HCC Tissues

For identifying the level of *MCM6* in HCC, we detected the *MCM6* expression in HCC tissues by IHC staining (Figure 7(a)). The result indicated that *MCM6* were obviously enhanced in HCC tissue compared to corresponding paracancer tissue, which were consistent with the previous bioinformatics results. Moreover, Kaplan-Meier survival analysis also indicated that *MCM6* was negatively correlated with the prognosis in HCC patients (Figure 7(b)), suggesting that *MCM6* might be a prognostic marker for HCC patients. Therefore, these results sufficient suggested that *MCM6* was significantly increased in HCC, and the high expression of *MCM6* showed a worse prognosis for HCC patients, suggesting that *MCM6* was a potential oncogene in HCC.

### 3.5. Notch Signaling Activation Is Critical for *MCM6*-Mediated Proliferation

Hyperproliferation is a hallmark feature of cancer. To elucidate the association between cell proliferation and *MCM6* expression, we performed MTT and colony formation analysis to confirm the proliferation ability in *MCM6* inhibition cells. This result showed that *MCM6* inhibition could significantly repress the proliferation ability for HepG2 and SNU-368 cell lines (Figures 7(c) and 7(d)). Moreover, GSEA analysis showed that *MCM6* was obviously enriched in the Notch signaling pathway (Figure 7(e)), which is closely correlated with cell proliferation in multiple cancer types. We further confirmed the expression of key factors involved in the Notch signaling pathway and EMT cascade by western blot, such as *E-cadherin*, *N-cadherin Notch1*, *Hey1*, and *Hes1* (Figure 7(f)). *MCM6* inhibition could significantly enhance the expression of *E-cadherin*, but repress the expression of N-cadherin, *Notch1*, *Hey1*, and *Hes1*, which suggested that *MCM6* inhibition could downregulate the proliferation ability of HCC cells via inactivating Notch pathway and EMT cascade.

## 4. Discussion

*MCM6*, a member of minichromosome maintenance proteins, has been demonstrated that it has a high level in HCC [10]. *MCM6* has multiple pathophysiological functions in carcinogenesis, especially in the hepatocarcinogenesis. Chen et al. found that *MCM6* knockdown could directly inhibit p53-binding protein 1 (*53BP1*) foci formation and chromatin fraction in response to DNA damage, indicating that *MCM6* was not just a DNA replication regulator [11]. Liu and his colleagues also revealed that *MCM6* could obviously promote migration and invasion ability via activating *MEK/ERK* signaling pathway to induce EMT cascades [10]. However, there are few studies mentioning the ancillary effects beyond DNA replication. And the ectopic expression of *MCM6* in the formation of HCC is still largely unknown. This study was based on the bioinformatics analysis of databases. After analysis of Oncomine, HCCDB, and TCGA databases, *MCM6* transcription and posttranscriptional levels were significantly upregulated in HCC. In subgroup analyses based on disease stage, tumor grade, age, gender, ethnicity, and body weight, the *MCM6* levels were significantly higher in HCC patients than in healthy people. Furthermore, the cBioPortal databases revealed that the frequencies of alterations of *MCM6* might be one reason for its ectopic expression and induce a low survival rate in HCC patients with *MCM6* alteration. The UALCAN databases also indicated that HCC patients with high expression of *MCM6* had a poorer survival rate.

*MCM6* is mainly involved in primary bile acid biosynthesis, valine, leucine and isoleucine degradation, arginine biosynthesis, DNA replication, fatty acid degradation, and homologous recombination by mining-related functional networks through the KEGG pathway. As we know, *MCM6* is a DNA replication license regulator that plays a key role in the cell cycle progression. It has been reported that *MCM6* could interact with other MCM proteins (*MCM2*, *MCM3*, *MCM4*, *MCM5*, *and MCM7*) to assemble into MCM complex, regulating the DNA replication to accelerate cell cycle [6]. However, the effect of *MCM6* on cell metabolism, such as primary bile acid, amino acid, and fatty acid, remains unclear [13]. We speculate that *MCM6*, like a molecular switch, has a divergence in these critical nodes, with one branch forming MCM complex to directly accelerate DNA replication and another branch regulating cell metabolism to provide the necessary materials and energy in DNA replication.

Furthermore, we found several genes associated with *MCM6*. The level of *NDUFAF1*, *LDHD*, and *SERPING1* were negatively correlated with *MCM6* expression levels. *NDUFAF1*, also known as NADH ubiquinone oxidoreductase complex assembly factor 1, is an essential assembly mitochondrial protein for the stability of complex I (NADH: ubiquinone oxidoreductase), which may play a key role in energy metabolism [14]. *LDHD*, lactate dehydrogenase D, is responsible for human D-lactate metabolism [15]. The upregulation of D-lactate metabolism is deemed as a consequence of the metabolic switch to aerobic glycolysis [16]. However, the function of *LDHD* in HCC progression is still unclear. *SERPING1*, serpin family G member 1, plays a key role in hereditary angioneurotic edema by inhibiting the classical complement pathway activation [17], which decreased in breast cancer [18], prostate cancer [19], and lung cancer [20]. Therefore, our analysis showed that *MCM6* might repress the tricarboxylic acid cycle by inhibiting the expression of *NDUFAF1*, inhibit aerobic glycolysis by inhibiting the expression of *LDHD*, and regulate the classical complement pathway activation by regulating the expression of *SERPING1*. *DTL*, *ZWINT*, and *MCM2* were increased with *MCM6* in HCC. *DTL* (denticleless E3 ubiquitin protein ligase homolog), also known as DNA replication factor 2, could mediate many cell cycle regulatory proteins levels to accelerate the cell cycle and maintain DNA repair and replication [21]. *ZWINT* (ZW10 interacting protein) interacted with ZW10, a key factor for spindle checkpoint control and chromosome motility, inhibited the chromosome bridge phenotype from interacting with sister chromatids [22]. *ZWINT* knockdown could attenuate mitotic arrest mediated by the microtubule inhibitor nocodazole, resulting in cell death [23]. *MCM2* could interact with *MCM3-7* to form a hexameric ring-shaped complex around DNA, which could promote DNA replication to accelerate the cell cycle [24]. Several previous studies indicated that *MCM2* could be an important biomarker of multiple cancer types, such as oral squamous cell carcinoma [25], cervical carcinoma [26], and medulloblastoma [27]. Hence, *MCM6* not only interact with *MCM2* to form a DNA replication license complex to directly activate DNA replication, but also interacts with *DTL* as well as *ZWINT* to accelerate the cell cycle. We also confirmed that *MCM6* was significantly upregulated in HCC samples, which was in accordance with previous studies [28, 29]. Moreover, we found that *MCM6* can interact with Notch pathway to enhance the proliferation level in HCC cells.

Notch pathway is a classical and important signaling in multiple cancer types, such as breast cancer, HCC, lung cancer, ovarian cancer, cervical cancer, gastric cancer, and renal carcinoma [30]. This signaling could also cross talk with other pathways, including PI3K/AKT, NF-*κ*B, integrin, and miRNAs, to significantly drive cell progression [31]. Previous study has indicated that Notch signaling is critical to cancer cell proliferation, apoptosis escaping, angiogenesis, EMT cascade, and stemness maintaining [32]. Because of Notch pathway is upregulated in HCC patients, the targeted treatment for anti-Notch pathway in HCC patients will need considerable on the upstream of Notch pathway, which are important to reduce the major side effects [33]. Our study indicated that MCM6 could activate the Notch pathway. The MCM6 might be a significant target for anti-Notch treatment in HCC patients.

## 5. Conclusion

This study indicates that *MCM6* is highly expressed in HCC compared to normal liver tissues and is correlated with multiple networks. *MCM6* is an excellent biomarker for predicting the prognosis of HCC. However, current research focuses on the role of *MCM6* in DNA replication. The role of *MCM6* in tumor metabolism is required to confirm the effect of *MCM6* on tumor metabolism and transcriptional regulation in HCC and other cancers. Moreover, *MCM6* is a carcinogenic role in activating Notch pathway to promote HCC cell proliferation, which may be a new therapeutic target for HCC patients.

## Figures and Tables

**Figure 1:** *MCM6* transcription in HCC. (a) *MCM6* level in cancer tissues vs. corresponding normal tissues by the Oncomine. (b) The transcriptional level of *MCM6* was analyzed in HCC among three studies by Oncomine. (c) *MCM6* level in the HCCDB database.

**Figure 2:** The transcription level of *MCM6* in HCC based on TCGA database. (a) *MCM6* gene level in multiple cancer types vs. corresponding normal tissues (TCGA). (b) Boxplot revealing *MCM6* level in normal people or HCC patients with cancer grade, (c) stage, (d) different ages, (e) gender, (f) ethnicity, and (g) weight.

**Figure 3:** The alterations and survival analysis of *MCM6* in HCC. (a) *MCM6* genetic alteration in AMC hepatology 2014 dataset, INSERM Nat Genet 2015 dataset, TCGA Firehose Legacy dataset. (b) OncoPrint of *MCM6* alterations in HCC. (c) The overall survival Kaplan-Meier estimate between HCC patients with and without *MCM6* alterations. (d) The disease/progression-free Kaplan-Meier estimate between HCC patients with and without *MCM6* alterations. (e) High level of *MCM6* was correlated with worse prognosis.

**Figure 4:** The DEGs associated with *MCM6* in HCC. Heat maps was used to analyze these DEGs negatively (a) and positively (b) correlated with *MCM6* in HCC. (c) Volcano plot was used to analyze these DEGs correlated with *MCM6* in HCC.

**Figure 5:** Identification of the association of *MCM6* and the top 3 DEGs based on TCGA. (a–c) The top three negative correlation genes (*NDUFAF1*, *LDHD*, and *SERPING1*) with *MCM6*. (d–f) The top three positive correlation genes (*DTL*, *ZWINT*, and *MCM2*) with *MCM6.*

**Figure 6:** GO and KEGG analysis of *MCM6* and these DEGs in HCC. (a) Biological processes. (b) Cellular components. (c) Molecular functions. (d) KEGG pathway analysis.

**Figure 7:** Identification of *MCM6* expression, function, and mechanism in HCC. (a) IHC staining of *MCM6* expression in HCC and corresponding paracancer tissues from 30 HCC patients. T: tumor; N: nontumor tissues. (b) Kaplan–Meier survival analysis for HCC patients with high or low *MCM6* expression based on KM-plot database (*P* < 0.05, log-rank test). (c) The MTT analysis and (d) clone formation analysis among HepG2 and SNU-368 cell lines with vector, *MCM6* shRNA or not. (e) The GSEA for *MCM6* in KEGG_Notch_signaling_pathway. (f) The expression of *MCM6*, *N-cadherin, E-cadherin*, *NCID*, *Notch1*, *Hey1*, and *Hes1* in HepG2 and SNU-368 cell lines with vector, *MCM6* shRNA or not. ∗∗*P* < 0.01 and ∗∗∗*P* < 0.001.

## Data Availability

The data used to support the findings of this study are available from the corresponding author upon request.
